# LncRNA SOX2-OTinhibitionprotects against myocardialischemia/reperfusion-inducedinjury via themicroRNA-186-5p (miR-186-5p)/Yin Yang 1 (YY1)pathway

**DOI:** 10.1080/21655979.2021.2000229

**Published:** 2021-12-30

**Authors:** Pengjie Yang, Kun Liang, Weisong Wang, Dehua Zhou, Yuan Chen, Xueyan Jiang, Rong Fu, Benben Zhu, Xuefeng Lin

**Affiliations:** a Department of Thoracic Surgery, Affiliated People’s Hospital of Inner Mongolia Medical University; b Geriatric Medical Center, Inner Mongolia People’s Hospital, Hohhot, China; c Department of Dispensary, Affiliated Hospital of Inner Mongolia Medical University; d Department of Emergency, People’s Hospital of Inner Mongolia Autonomous Region; e Department of Pharmacy, Affiliated People’s Hospital of Inner Mongolia Medical University, Hohhot, P.R.China; f Department of Cardiovascular Medicine, First Affiliated Hospital of Baotou Medical College, Baotou, P.R.China

**Keywords:** Myocardial ischemia/reperfusion-induced injury, SOX2-OT, miR-186-5p, YY1

## Abstract

Long noncoding RNAs (lncRNAs) exert essential effects in regulating myocardial ischemia/reperfusion (MI/R)-induced injury. This work intended to explore the functions of lncRNA SOX2-OT and its regulatory mechanism within MI/R-induced injury. In this study, gene expression was determined by RT-qPCR. Western blotting was applied for the detection of protein levels. Pro-inflammatory cytokine concentrations, cardiomyocyte viability, and apoptosis were detected via ELISA, CCK-8 and flow cytometry. In the in vitro model, SOX2-OT and YY1 were both upregulated, while miR-186-5p was downregulated. SOX2-OT knockdown attenuated oxygen-glucose deprivation/reoxygenation (OGD/R)-induced cardiomyocyte dysregulation through relieving inflammation, promoting proliferation, and reducing apoptosis in OGD/R-treated H2C9 cells. SOX2-OT positively regulated YY1 expression via miR-186-5p. Moreover, miR-186-5p inhibition or YY1 upregulation abolished the effects of SOX2-OT blocking on the inflammatory responses, proliferation, and apoptosis of OGD/R-challenged H2C9 cells. In conclusion, our results, for the first time, demonstrated that SOX2-OT inhibition attenuated MI/R injury in vitro via regulating the miR-186-5p/YY1 axis, offering potential therapeutic targets for MI/R injury treatment.

## Introduction

Acute myocardial infarction (AMI), owing to deficient blood flow to cardiac tissue, poses a threat to human health as a primary cause for mortality in the world [1]. At present, percutaneous coronary intervention (PCI) is a major therapeutic method for AMI treatment [2]; contradictorily, PCI may also lead to myocardial ischemia/reperfusion (MI/R) injury since sudden blood flow restoration could cause secondary damages to the myocardial tissues injured in AMI [3]. Approximately, 50% of AMI patients suffer from myocardium necrosis due to MI/R injury [4]. Hence, prevention and treatment of MI/R-induced injury are of significance for the improvement of clinical outcomes in AMI patients.

The mechanisms of MI/R injury may involve multiple pathological and physiological processes, including oxidative stress, inflammatory response, cell proliferation, and cell apoptosis [5,6]. MI/R injury can induce cell membrane destruction, leading to creatine kinase-muscle/brain (CK-MB) and lactate dehydrogenase (LDH) leakage [7]. Sterile inflammatory responses caused by MI/R injury may also lead to further injury and even contribute to increment in the final size of myocardial infarct [8]. Therefore, molecules could be implicated in MI/R injury via regulating these physiopathological pathways.

Long non-coding RNA (LncRNA) is a class of non-coding transcripts (over 200 nucleotides in length) with essential regulatory effects on biological processes [9]. So far, a great number of lncRNAs have been ascertained as vital regulators in MI/R injuries. For instance, lncRNA Oip5-as1 activates the SIRT1/AMPK/PGC1α cascade via miR-29a, thereby alleviating MI/R injury [10]. LncRNA PEAMIR expedited MI/R injury via miR-29b-3p [11]. Besides, lncRNA GAS5 aggravates MI/R injury via the miR-137/serpina3 axis [12]. A former report from Greco et al. identified lncRNA SOX2-OT as an upregulated lncRNA in ischemic heart failure [13]. Nevertheless, the role and potential mechanisms of SOX2-OT in MI/R injury are still obscure.

In this work, we intended to explore the role of SOX2-OT in MI/R injury and the specific mechanism by which SOX2-OT affects MI/R injury in vitro. First of all, an in vitro OGD/R-induced H2C9 cell model was established. Via functional experiments on the cell model of MI/R injury, we found SOX2-OT could promoted OGD/R-induced H2C9 cell dysfunction, thus providing promising therapeutic targets for the treatment of MI/R injury.

## Materials and methods

### Cell culture

As per the standard protocols, murine embryonic cardiomyocyte cell line (H2C9) bought from BeNa Culture Collection (Beijing, China) was cultivated in DMEM in an incubator (95% air+5% CO_2_) at 37°C for 24 h before further treatment.

### Cell transfection

MiR-186-5p mimics, miR-186-5p inhibitor, their negative controls (NC mimics and NC inhibitor), siRNA against SOX2-OT (si-SOX2-OT), negative control (si-NC), pcDNA3.1/SOX2-OT (SOX2-OT), pcDNA3.1/YY1 (YY1), and empty pcDNA3.1 (Vector) obtained from GenePharma were transfected into H2C9 cardiomyocytes via Lipofectamine 2000 (Invitrogen, USA).

### Establishment of oxygen-glucose deprivation/reoxygenation (OGD/R) cell model

To construct an OGD/R cell model, H2C9 cardiomyocytes were seeded into glucose-free DMEM and cultivated in the atmosphere containing 95% N_2_ and 5% CO_2_ for 4 h at 37°C. Thereafter, the H2C9 cells were transferred to fresh normal DMEM containing 4.5 mg/mL glucose and cultured in the regular incubator (95% air+5% CO_2_) at 37°C for 24 h. Untreated H2C9 cardiomyocytes were used as the Control group [14].

### RT-qPCR

Via TRIzol Reagent (Invitrogen, Carlsbad, CA), total RNAs were extracted from cells. For lncRNA and mRNA, cDNA was synthesized by reversely transcribing RNA via PrimeScript™ RT Reagent Kit (Takara; Kusatsu, Japan); then, qPCR was performed with TB Green™ Premix Ex Taq™ (Takara; Kusatsu, Japan), with GAPDH as the internal reference. Considering miRNA, cDNA was synthesized by reversely transcribing RNA via miRNA 1st Strand cDNA Synthesis Kit (GeneCopeia; Guangzhou, China); then, qPCR was conducted by SYBR Green PCR Master Mix (Applied Biosystems), with U6 as the internal reference. The quality and quantity of total RNA was assessed with a NanoDrop 1000 spectrophotometer (Thermo Fisher Scientific, Inc.). The following thermocycling parameters were applied for qPCR: 95°C for 30 seconds, followed by 30 cycles for denaturation at 95°C for 5 seconds, annealing at 60°C for 30 seconds, and extension at 72°C for 30 seconds. Finally, Relative gene expression levels were calculated by 2^−ΔΔCt^ method. All the primers adopted were as follows: SOX2-OT forward (F): 5ʹ-GCTCGTGGCTTAGGAGATTG-3ʹ and reverse (R): 5ʹ-CTGGCAAAGCATGAGGAACT-3ʹ; YY1 F: 5ʹ-ATCTATCCGCCGTGTGGGA-3ʹ and R: 5ʹ-ATGGCGGCTTGAATTTCTCG-3ʹ; GAPDH F: 5ʹ-CAGGAGGCATTGCTGATGAT-3ʹ and R: 5ʹ-GAAGGCTGGGGCTCATTT-3ʹ; miR-186-5p F: 5ʹ-CGCCGCAAAGAATTCTCCTTT-3ʹ and R: 5ʹ-GTGCAGGGTCCGAGGT-3ʹ; U6 F: 5ʹ-TTCACGAATTTGCGTGTCATC-3ʹ and R: 5ʹ-AAAATATGGAACGC-3ʹ.

### ELISA

The concentrations of pro-inflammatory factors, such as interleukin-1β (IL-1β), interleukin-6 (IL-6), and tumor necrosis factor-α (TNF-α) were detected with the ELISA kit (BD Biosciences) as per the manufacturer’s instructions [15].

### CCK-8

The cell proliferative capability was detected by CCK-8 assay. Briefly, H2C9 cardiomyocytes (1 × 10^4^ cells/well) were plated into a 96-well plate. Following respective treatment, 10 μL CCK-8 solution was added to each well. Thereafter, H2C9 cells were cultured at 37°C for another 2 h. The optical density (OD) was detected with a microplate reader (ThermoFisher Scientific, USA) [16].

### Flow cytometry

To analyze cardiomyocyte apoptosis, Annexin V-FITC/PI Apoptosis Detection Kit (YEASEN, Shanghai) was applied. Briefly, H2C9 cells were re-suspended in 100 μL binding buffer supplemented with 5 μL Annexin V-FITC and 10 μL PI reagent and then cultured in darkness for 10 min. Through flow cytometry (BD FACS Canto II, USA), the apoptotic cells were detected [17].

### Western blotting

With RIPA protein extraction reagent, protein homogenates were extracted from cells. Then, the protein homogenates were separated into equal amounts by SDS-PAGE and transferred to PVDF membranes (Millipore). Then, the membranes were cultured with primary antibodies against YY1, and apoptosis-associated factors (Bcl-2 and cleaved caspase-3) at 4°C overnight after being blocked in 5% nonfat milk. Thereafter, the membranes were cultured with secondary antibodies at room temperature for 2 h. At last, ECL Western blotting substrate (Pierce) was applied for visualization of protein bands [18].

### Dual-luciferase reporter assay

The synthesized SOX2-OT or YY1 wild-type/mutant-type reporter vectors (SOX2-OT/WT or SOX2-OT/MUT; YY1/WT or YY1/MUT) (Ribobio, China) were cot-transfected into H2C9 cardiomyocytes together with NC mimics or miR-186-5p mimics for 24 h at room temperature. Afterward, Dual-luciferase Reporter Assay System (Promega) was applied for luciferase activity assessment [19].

## Statistical analysis

In this work, data were shown as mean±SD. GraphPad 6.0 software was used to carry out all the statistical analyses. The normality of the distribution was checked by Shapiro-Wilk test. Comparison between several groups or two groups among was performed via one-way ANOVA or Student’s t-test. Any difference with *P*-value < 0.05 was deemed significant in statistics.

## Results

Herein, we intended to investigate the role and specific regulatory mechanism of SOX2-OT in MI/R injury via an in vitro OGD/R cell model established on H2C9 cells. Through a series of in vitro assays, we discovered that SOX2-OT was highly expressed in OGD/R-treated H2C9 cells and impaired the functions of H2C9 cells via the miR-186-5p/YY1 axis, offering novel target genes for the diagnosis and treatment of MI/R injury.

### SOX2-OT is highly expressed in OGD/R-treated cardiomyocytes and aggravates OGD/R-triggered cardiomyocyte dysfunction

To investigate the role of SOX2-OT in MI/R-induced injury, we firstly constructed an OGD/R-induced cell model with the embryonic rat cardiomyocyte cell line (H2C9). As indicated by RT-qPCR, SOX2-OT expression was notably boosted in OGD/R-treated H2C9 cardiomyocytes (Figure 1(a)). Therefore, it was speculated that SOX2-OT participated in the MI/R progression.

**Figure 1.** SOX2-OT is highly expressed in OGD/R-treated cardiomyocytes and aggravates OGD/R-triggered cardiomyocyte dysfunction. (a) SOX2-OT expression in H9C2 cardiomyocytes from Control group and OGD/R group was determined via RT-qPCR. (b) OGD/R-induced H9C2 cardiomyocytes were transfected by si-NC or si-SOX2-OT, respectively. RT-qPCR verified SOX2-OT knockdown efficiency in OGD/R-induced H9C2 cardiomyocytes. (c-e) The pro-inflammatory cytokine (IL-1β, IL-6, and TNF-α) levels were assessed via ELISA in the Control group, OGD/R group, OGD/R+ si-NC group, or OGD/R+ si-SOX2-OT group. F) CCK-8 was utilized to detect cell viability in each group. (g) Flow cytometry was utilized to detect cell apoptosis in each group. (h) Western blotting assay was applied to detect the levels of apoptosis-related proteins (Bcl-2 and cleaved caspase-3). *P < 0.05; **P < 0.01; ***P < 0.001.

To inquire into the function of SOX2-OT in OGD/R-treated cardiomyocytes, SOX2-OT was firstly knocked down in OGD/R-induced H2C9 cells. RT-qPCR assay verified SOX2-OT knockdown efficiency (Figure 1(b)). As determined through ELISA assay, the pro-inflammatory factor (TNF-α, IL-1β, and IL-6) levels were apparently elevated after exposure to OGD/R and decreased after blocking SOX2-OT (Figure 1(c-e)). CCK-8 assay manifested that OGD/R treatment apparently decreased H2C9 cell viability, relative to the control group; while SOX2-OT silencing significantly enhanced the viability of OGD/R-treated H2C9 cardiomyocytes (figure 1(f)). In addition, flow cytometry results revealed that SOX2-OT depletion remarkably reduced OGD/R-induced H2C9 cell apoptosis (Figure 1(g)). In line with the above data, western blotting assay showed that OGD/R treatment distinctly reduced the Bcl-2 level but increased cleaved caspase-3 level in H2C9 cardiomyocytes, while SOX2-OT knockdown visibly reversed such regulatory effects on these apoptosis-related proteins caused by OGD/R treatment (Figure 1(h)). Taken together, downregulation of SOX2-OT might relieve cardiomyocyte dysfunction induced by OGD/R.

### SOX2-OT binds to miR-186-5p

To understand the molecular mechanism by which SOX2-OT regulates MI/R injury, StarBase website was applied to predict target miRNAs for SOX2-OT. Among the miRNAs predicted, miR-186-5p was found to play vital roles in regulating apoptosis of cardiomyocytes induced by high glucose or ethanol. Moreover, miR-186-5p abundance was lowly expressed in OGD/R-challenged H2C9 cardiomyocytes (Figure 2(a)). Therefore, miR-186-5p was used for further investigation. A binding site was predicted between miR-186-5p and SOX2-OT (Figure 2(b)). Then, miR-186-5p was overexpressed in OGD/R-induced H2C9 cells (Figure 2(c)). The dual-luciferase assay exhibited that miR-186-5p addition prominently reduced the luciferase activity of SOX2-OT-WT, while exerted almost no influence on the luciferase activity of SOX2-OT-MUT (Figure 2(d)). As shown in Figure 2(e), SOX2-OT was also overexpressed in OGD/R-treated H2C9 cells. Next, SOX2-OT inhibition significantly upregulated miR-186-5p expression, whereas SOX2-OT overexpression markedly decreased miR-186-5p abundance in OGD/R-induced H2C9 cells (figure 2(f)). Hence, SOX2-OT negatively modulated miR-186-5p in OGD/R cardiomyocyte model.

**Figure 2.** SOX2-OT binds to miR-186-5p. (a) MiR-186-5p expression in H9C2 cardiomyocytes from Control group and OGD/R group was determined via RT-qPCR. (b) The potential targeting region was predicted by StarBase website. (c) OGD/R-induced H9C2 cardiomyocytes were transfected by NC mimics or miR-186-5p mimics, respectively. RT-qPCR verified miR-186-5p overexpression efficiency in OGD/R-induced H9C2 cardiomyocytes. (d) Luciferase assay was performed to verify whether miR-186-5p targeted SOX2-OT in OGD/R-induced H9C2 cardiomyocytes. (e) OGD/R-induced H9C2 cardiomyocytes were transfected by Vector or SOX2-OT, respectively. RT-qPCR verified SOX2-OT overexpression efficiency in OGD/R-induced H9C2 cardiomyocytes. (f) MiR-186-5p expression in OGD/R-induced H9C2 transfected by si-NC, si-SOX2-OT, Vector, or SOX2-OT was determined via RT-qPCR. *P < 0.05; **P < 0.01.

### SOX2-OT regulates OGD/R-treated cardiomyocyte injury by targeting miR-186-5p

To further verify whether miR-186-5p is involved in the OGD/R-induced H2C9 cellular processes regulated by SOX2-OT, a series of rescue experiments were conducted. First of all, miR-186-5p expression was knocked down in OGD/R-induced H2C9 cells (Figure 3(a)). As indicated by ELISA assay, SOX2-OT knockdown decreased IL-1β, IL-6, and TNF-α levels in OGD/R-induced H2C9 cells, which could be partially abrogated by miR-186-5p inhibition (Figure 3(b-d)). As shown in CCK-8 results, the proliferation of OGD/R-treated H2C9 cells was substantially enhanced by SOX2-OT knockdown, which could be partly abrogated by miR-186-5p suppression (Figure 3(e)). The results of flow cytometry analysis showed that SOX2-OT inhibition reduced the apoptotic rate of H2C9 cells induced by OGD/R, while miR-186-5p repression partially abolished the effect of SOX2-OT silencing (figure 3(f)). Moreover, such variations in H2C9 cell apoptosis were also manifested as the altered protein levels of apoptotic markers (Figure 3(g)). To sum up, SOX2-OT aggravated the cardiomyocyte dysfunction caused by OGD/R treatment as a ceRNA for miR-186-5p.

**Figure 3.** SOX2-OT regulates OGD/R-treated cardiomyocyte injury by targeting miR-186-5p. (a) OGD/R-induced H9C2 cardiomyocytes were transfected by NC inhibitor or miR-186-5p inhibitor, respectively. RT-qPCR verified miR-186-5p knockdown efficiency in OGD/R-induced H9C2 cardiomyocytes. (b-d) The pro-inflammatory cytokine (IL-1β, IL-6, and TNF-α) levels were assessed via ELISA in OGD/R-induced H9C2 cardiomyocytes transfected with si-NC, si-SOX2-OT, si-SOX2-OT+NC inhibitor, or si-SOX2-OT+miR-186-5p inhibitor. (e) CCK-8 was utilized to detect cell viability in each group. (f) Flow cytometry was utilized to detect cell apoptosis in each group. (g) Western blotting assay was applied to detect the levels of apoptosis-related proteins (Bcl-2 and cleaved caspase-3). *P < 0.05; **P < 0.01.

### YY1 is directly targeted by miR-186-5p in OGD/R-induced cardiomyocytes

To further explore the downstream mechanism of SOX2-OT/miR-186-5p cascade in MI/R, target genes for miR-186-5p were predicted by 4 miRNA databases (microT, miRanda, PicTar, and TargetScan) under certain condition (CLIP Data: strict stringency ≥5). 7 candidate genes (CSNK2A1, EED, YY1, UBE2R2, PSME3, NCBP2, and TEAD1) were screened (Figure 4(a)). Among them, YY1 is upregulated in human heart failure [20]. In addition, YY1 enrichment was upregulated in OGD/R-treated H2C9 cardiomyocytes (Figure 4(b,c)). Therefore, YY1 was selected for further investigation. StarBase website provides the binding site between YY1 and miR-186-5p (Figure 4(d)). Next, luciferase assay confirmed that miR-186-5p downregulated the luciferase activity in OGD/R-induced H2C9 cardiomyocytes co-transfected with YY1-WT, rather than YY1-MUT (Figure 4(e)), suggesting that miR-186-5p interacts with YY1 in OGD/R-induced H2C9 cells. Western blotting assays indicated that miR-186-5p suppression increased the mRNA and protein levels of YY1, while such an increase could be partially offset by SOX2-OT blocking (figure 4(f,g)). These results indicated that SOX2-OT positively regulated YY1 via targeting miR-186-5p.

**Figure 4.** YY1 is directly targeted by MiR-186-5p in OGD/R-induced cardiomyocytes. (a) Venn diagram of candidate mRNAs for miR-186-5p predicted by microT, miRanda, PicTar, and TargetScan. (b and c) YY1 mRNA and protein levels in H9C2 cardiomyocytes from Control group and OGD/R group were determined via RT-qPCR and Western blotting. (d) The potential targeting region was predicted by StarBase website. (e) Luciferase assay was performed to verify whether miR-186-5p targeted YY1 in OGD/R-induced H9C2 cardiomyocytes. (f and g) YY1 mRNA and protein levels in OGD/R-induced H9C2 transfected by NC inhibitor, miR-186-5p inhibitor, miR-186-5p inhibitor+si-NC, or miR-186-5p inhibitor+si-SOX2-OT were determined via RT-qPCR and Western blotting. *P < 0.05; **P < 0.01.

### SOX2-OT depletion exerts protective effects by regulating YY1 expression

To further probe about whether YY1 is implicated in the impact of SOX2-OT on OGD/R-induced H2C9 cells, YY1 overexpression was performed in OGD/R-induced H2C9 cardiomyocytes (Figure 5(a,b)). It was found that YY1 mRNA and protein levels were both decreased after SOX2-OT silencing and partially recovered after YY1 upregulation (Figure 5(c,d)). Besides, YY1 overexpression partly neutralized the influence of SOX2-OT silencing on the pro-inflammatory cytokine levels, cell viability, apoptosis, as well as levels of apoptosis-associated proteins (Figure 5(e-j)). Collectively, SOX2-OT knockdown exerts protective effects on OGD/R-challenged cardiomyocytes via regulating YY1.

**Figure 5.** SOX2-OT depletion exerts protective effects by regulating YY1 expression. (a and b) OGD/R-induced H9C2 cardiomyocytes were transfected by Vector or YY1, respectively. RT-qPCR and Western blotting assays verified YY1 overexpression efficiency in OGD/R-induced H9C2 cardiomyocytes. (c and d) YY1 mRNA and protein levels in OGD/R-induced H9C2 transfected by si-NC, si-SOX2-OT, Vector, or YY1 were determined via RT-qPCR and Western blotting. (e-g) The pro-inflammatory cytokine (IL-1β, IL-6, and TNF-α) levels were assessed via ELISA in OGD/R-induced H9C2 cardiomyocytes transfected with si-NC, si-SOX2-OT, si-SOX2-OT+Vector, or si-SOX2-OT+YY1. (h) CCK-8 was utilized to detect cell viability in each group. (i) Flow cytometry was utilized to detect cell apoptosis in each group. (j) Western blotting assay was applied to detect the levels of apoptosis-related proteins (Bcl-2 and cleaved caspase-3). *P < 0.05; **P < 0.01.

## Discussion

As suggested by previous studies, lncRNAs are emerging regulators in cardiovascular diseases, including MI/R injury [21]. For example, Luo et al. demonstrated that lncRNA H19 silencing relieves MI/R injury by regulating PPARα via miR-675 [22]. Zhao et al. revealed that lncRNA Gm4419 aggravates MI/R injury by regulating TRAF3 via miR-682 [23]. It was uncovered by Sun et al. that lncRNA HOTAIR knockdown protected against MI/R injury via the miR-126/SRSF1 pathway [24]. LncRNA SOX2-OT has been reported to participate in a variety of cellular processes, including apoptosis, inflammatory response, and proliferation [25–27]. SOX2-OT also plays a vital role in cardiovascular diseases. To cite an instance, Gu et al. elaborated that SOX2-OT facilitated inflammation and apoptosis in ischemic heart failure by regulating TRAF6 via miR-455-3p [25]. As elucidated in a report from Yang et al., SOX2-OT aggravated myocardial infarction through the miR-27a-3p/TGFBR1 pathway [28]. Similarly, Tu et al. found that SOX2-OT exacerbated ischemia-induced heart failure in a murine model [29]. In addition, SOX2-OT inhibition could alleviate cerebral I/R injury via the miR-135a-5p/NR3C2 pathway [30], indicating its promoting role in I/R injuries. In line with the above studies, we demonstrated that SOX2-OT expression was lifted in OGD/R-treated H2C9 cells. Besides, SOX2-OT knockdown reduced the pro-inflammatory cytokine levels, facilitated H2C9 cardiomyocyte proliferation, and inhibited H2C9 cardiomyocyte apoptosis. It was also found that SOX2-OT silencing reduced the cleaved caspase-3 level but upregulated the Bcl-2 level in H2C9 cells. Our findings suggested that SOX2-OT plays a vital role during MI/R.

LncRNAs exert crucial effects in cellular processes by regulating mRNA expressions as competing endogenous RNAs (ceRNAs) for microRNAs (miRNA) [31]. MiR-186-5p could relieve I/R-induced injury in spinal cord by reducing inflammation [32]. Besides, the cardioprotective role of miR-186-5p has also been demonstrated in numerous studies. As an example, Ren et al. revealed that miR-186-5p protected against PPF-induced cardiac cytotoxicity [33]. Liu et al. uncovered that miR-186-5p reduced cardiomyocyte apoptosis induced by high glucose [34]. In this work, miR-186-5p was verified as a target for SOX2-OT through bioinformatic tools and dual-luciferase assay. MiR-186-5p abundance was lowly expressed in OGD/R-treated H2C9 cardiomyocytes. MiR-186-5p inhibition reversed the effects of SOX2-OT inhibition on the inflammatory responses, proliferation, and apoptosis of OGD/R-challenged H2C9 cells. Consistent with the above studies, our results suggested that miR-186-5p attenuated inflammation, promoted proliferation, and reduce apoptosis in OGD/R-treated H2C9 cells. Therefore, SOX2-OT aggravated MI/R injury in vitro via negatively regulating miR-186-5p.

Yin Yang 1 (YY1) plays complex regulatory roles in cardiovascular diseases. YY1 protected against cardiac fibrosis and dilated cardiomyopathy via targeting BMP7 and CTGF [35]. However, isoproterenol treatment upregulated YY1 and inhibited CuZn-SOD, thus inducing oxidative stress and apoptosis in H9C2 cardiomyocytes [36]. Besides, YY1 also exacerbates I/R-induced cerebral and hepatic injuries [37,38], suggesting its promoting role in the progression of I/R-induced injury. Herein, YY1 was verified as a downstream target gene for miR-186-5p. YY1 expression was elevated in OGD/R-treated H2C9 cardiomyocytes. SOX2-OT positively regulated YY1 expression as a ceRNA for miR-186-5p. In consonance with previous research results, YY1 upregulation partly neutralized the protective effects of SOX2-OT knockdown on OGD/R-challenged H2C9 cells via regulating inflammatory responses, proliferation, and apoptosis in H2C9. Hence, SOX2-OT aggravated the dysfunction of OGD/R-treated cardiomyocytes by modulating YY1 via miR-186-5p.

## Conclusion

In summary, this study for the first time demonstrated that SOX2-OT promoted OGD/R-induced cardiomyocyte dysfunction by aggravating inflammation, inhibiting cardiomyocyte proliferation, and increasing cardiomyocyte apoptosis via upregulating YY1 expression through interaction with miR-186-5p. Our findings indicated that SOX2-OT might be a new biomarker for the development and progression of MI/R injury, which could contribute to the research on the diagnosis and treatment of MI/R injury.
